# Overexpression of microRNA-195-5p reduces cisplatin resistance and angiogenesis in ovarian cancer by inhibiting the PSAT1-dependent GSK3β/β-catenin signaling pathway

This article has been retracted.

**DOI:** 10.1186/s12967-019-1932-1

**Published:** 2019-06-06

**Authors:** Jun Dai, Rujia Wei, Peihai Zhang, Beihua Kong

**Affiliations:** 1 Department of Gynecology and Obstetrics, Qilu Hospital of Shandong University, No. 107, Wenhua West Road, Jinan, 250012 Shandong People’s Republic of China; 2 School of Life Sciences, Liaocheng University, Liaocheng, 252000 People’s Republic of China; 3 Department of Gynecology and Obstetrics, Qilu Hospital of Shandong University (Qingdao Hospital District), No. 758, Hefei Road, Shibei District, Qingdao, 266035 Shandong People’s Republic of China

**Keywords:** MicroRNA-195-5p, Phosphoserine aminotransferase 1, Glycogen synthase kinase-3β/β-catenin signaling pathway, Ovarian cancer, Angiogenesis, Cisplatin resistance

## Abstract

**Background:**

Ovarian cancer (OC) is one of the leading causes for cancer-related deaths among women. MicroRNAs (miRs) have been proved to be vital to the development and progression of OC. Hence, the study aims to evaluate the ability of miR-195-5p affecting cisplatin (DDP) resistance and angiogenesis in OC and the underlying mechanism.

**Methods:**

MiRs that could target phosphoserine aminotransferase 1 (PSAT1), a differentially expressed gene in OC, were predicted by miRNA-mRNA prediction websites. The expression patterns of miR-195-5p in the OC tissues and cells were determined using RNA quantification assay. The role of miR-195-5p in OC was evaluated by determining DDP resistance, apoptosis and angiogenesis of OC cells after up-regulating or down-regulating miR-195-5p or PSAT1, or blocking the glycogen synthase kinase-3β (GSK3β)/β-catenin signaling pathway. Animal experiment was conducted to explore the effect of miR-195-5p on resistance to DDP and angiogenesis.

**Result:**

MiR-195-5p directly targeted PSAT1 and down-regulated its expression. The expression of miR-195-5p was lower while that of PSAT1 was higher in OC tissues than in adjacent normal tissues. When miR-195-5p was over-expressed or PSAT1 was silenced, the expression of HIF-1α, VEGF, PSAT1, β-catenin as well as the extent of GSK3β phosphorylation was reduced, the angiogenesis and resistance to DDP was diminished and apoptosis was promoted both in vitro and in vivo. The inhibition of GSK3β/β-catenin signaling pathway was involved in the regulation process.

**Conclusion:**

Over-expression of miR-195-5p reduced angiogenesis and DDP resistance in OC, which provides a potential therapeutic target for the treatment of OC.

## Background

Ovarian cancer (OC) is the 5th leading cause of cancer-related deaths among female with over 230,000 newly diagnosed cases every year [1, 2]. Unfortunately, the 5-year overall survival rate of patients suffering OC remains to be 30% [3]. There are three major types of OC including sex cord stromal, germ cell and epithelial tumors, among which epithelial ovarian cancer (EOC) represents around 90% of all OC occurrence accompanied by high mortality [4]. Ovarian carcinogenesis is associated with exposure to increased gonadotropins, continuous ovulation, inflammatory cytokines and sex-steroid hormones [5]. Currently, a combination therapy of platinum-based chemotherapy and optical cytoreductive surgery is widely used as the standard treatment for initial stage OC patients [6]. During platinum-based chemotherapy, cisplatin (DDP) is regarded as the first choice among chemotherapy drugs for OC treatment [7]. However, the survival rate of OC patients remains to be gloomy due to the recurrence and growing resistance to chemotherapy [8]. Therefore, a new therapeutic target is necessary to overcome the resistance to chemotherapy and improve the prognoses of OC patients.

Phosphoserine aminotransferase 1 (PSAT1), one of the serine synthesis related enzymes, which is highly expressed in various tissues [9]. In addition, PSAT1 has been proved to function as an oncogene, involved in tumor metastasis and development [10]. It is well-known that microRNAs (miRs) are small noncoding RNAs which possess the potential to typically repress the post-transcriptional level of messenger RNAs (mRNAs), thus regulating genes associated with cellular processes [11]. In the current study, we observed that PSAT1 was the target gene of miR-195-5p predicted by miRNA-mRNA relationship prediction websites. MiRs are involved in the progression of epithelial OC and exert regulatory effects on OC cell line characteristics [12]. Furthermore, miR-195-5p has been demonstrated to be involved in the regulation of numerous cancers and serves as a potential therapeutic target for the treatment of colorectal cancer (CRC) [13]. Moreover, miR-489 was revealed to repress the cell growth and DDP resistance while accelerating apoptosis in OC [14]. Similarly, miR-3646 facilitates docetaxel resistance through Glycogen synthase kinase-3β (GSK3β)/β-catenin signaling pathway in breast cancer cells [15]. Meanwhile, the motility of OC cells can be suppressed by huaier aqueous extract through the AKT/GSK3β/β-catenin signaling pathway [16]. More importantly, PSAT1 was found to mediate cell cycle progression in breast cancer via regulation of the GSK3β/β-catenin signaling pathway [10]. Based on previous findings and prediction results from the current study, we propose a hypothesis that miR-195-5p might affect the development and progression of OC with the involvement of PSAT1 and the GSK3β/β-catenin signaling pathway. Therefore, the current study aims to investigate the underlying molecular mechanism of miR-195-5p, PSAT1 and GSK3β/β-catenin signaling pathway in angiogenesis and DDP resistance, hoping to provide more effective therapy strategies for the treatment of OC.

## Materials and methods

### Ethical statements

The experiment protocol was approved by the Ethics Committee and Institutional Animal Care and Use Committee of Qilu Hospital of Shandong University (Qingdao Hospital District). Signed informed consents were obtained from all participants and the experiments were conducted in line with the ethical principles of Declaration of Helsinki. All animal experimentation was carried out in strict accordance with the recommendations in the Guide for the Care and Use of Laboratory Animals of the National Institutes of Health.

### Microarray analysis

Firstly, 5 OC-related microarray data (GSE54388, GSE40595, GSE38666, GSE18520, and GSE14407) were retrieved from gene expression omnibus (GEO) database (https://www.ncbi.nlm.nih.gov/geo/), and were screened for the differentially expressed genes (DEGs). Detailed information of the microarray data is shown in Table 1. The Affy package of R software was applied for background correction and standardized pretreatment on gene expression data, while the limma package was utilized to screen the DEGs. The corrected *p* value was expressed as *adj.P.Val*. With the |log2foldchange (FC)| > 2.0 and *adj.P.Val* < 0.05 serving as the screening threshold, the histogram of DEGs was plotted. Then Jvenn (http://jvenn.toulouse.inra.fr/app/example.html) was used to compare DEGs among the five datasets. The DiGSeE disease gene search engine (http://210.107.182.61/geneSearch/) was employed to retrieve OC-related genes. The String database (https://string-db.org/) was utilized to provide protein–protein interaction (PPI) information [17], while the Cytoscape 3.6.0 software was used to extract DEGs and disease genes of OC to construct the PPI network [18]. Afterwards, the miRNA–mRNA relationship prediction websites, TargetScan (http://www.targetscan.org/vert_71/), mirDIP (http://ophid.utoronto.ca/mirDIP/), miRpath (http://lgmb.fmrp.usp.br/mirnapath/tools.php), microRNA (http://34.236.212.39/microrna/getGeneForm.do), DIANA (http://diana.imis.athena-innovation.gr/DianaTools/index.php?r=microT_CDS/index) and miRSearch (http://www.exiqon.com/microrna-target-prediction) were applied to predict miRs that could regulate PSAT1, and compare their prediction results.

**Table 1:** OC-related gene chip information

Accession	Platform	Organism	Sample
GSE54388	GPL570	Homo sapiens	6 normal human ovarian surface epithelium and 16 serous ovarian cancer tumor epithelial
GSE40595	GPL570	Homo sapiens	6 normal ovarian surface epithelium samples and 32 samples of epithelial component from high grade serous ovarian cancer patients
GSE38666	GPL570	Homo sapiens	12 normal ovarian surface epithelium and 18 ovarian cancer epithelium
GSE18520	GPL570	Homo sapiens	53 papillary serous ovarian adenocarcinoma tumor specimens and 10 normal ovarian surface epithelium
GSE14407	GPL570	Homo sapiens	12 healthy ovarian surface epithelia samples were compared to 12 serous ovarian cancer epithelia samples

*OC* ovarian cancer

### Study subjects

A total of 77 cases pathologically confirmed primary OC tissues and 25 cases of normal ovarian tissues were obtained from patients undergoing ovarian resection because of non-ovarian lesions at the Qilu Hospital of Shandong University (Qingdao Hospital District) between 2014 and 2016. All OC patients were undergoing surgery for the first time, and had not received radiotherapy, chemotherapy or immunotherapy prior to the operation. After the operation, some fresh tissue samples were stored in liquid nitrogen for 30 min, and then stored at − 80 °C in a refrigerator for further experimentation. Baseline characteristics of the enrolled patients are described in Table 2.

**Table 2:** Characteristics of the studied OC patients

Characteristics	n
Age	
> 50 years	42
≤ 50 years	35
FIGO pathological stage	
Well and moderate differentiation (G1 + G2)	37
Poor differentiation (G3)	40
FIGO clinical stage	
Stage I–II	49
Stage III	28
Lymph node metastasis	
Yes	50
No	27

*FIGO* International Federation of Gynecology and Obstetrics, *OC* ovarian cancer

### Dual-luciferase reporter gene assay

The HEK-293T cell line (purchased from the Cell Bank of Shanghai Institute of Cells, Chinese Academy of Science, Shanghai, China) was cultured in Dulbecco’s modified Eagle medium (DMEM) sugar medium. Once the cell confluence reached 80–90%, the cells were detached and passaged with 0.25% trypsin, and conventionally cultured in a humidified incubator with 5% CO_2_ in air at 37 °C. Then cells at the logarithmic phase of growth were selected for further experiments. The Targetscan.org website was utilized to analyze the target gene of miR-195-5p, while a dual-luciferase reporter gene assay was applied to verify whether PSAT1 was the direct target gene of miR-195-5p. The synthesized PSAT1 3′ untranslated region (3′ UTR) gene fragment was introduced into the pGL3-control (Promega Corporation, Madison, WI, Wisconsin, USA) by endonuclease sites *Xho*I and *Bam*HI. Complementary mutant (MUT) sites of seed sequence were designed based on the PSAT1 wild-type (WT) sequence, and then the target fragment was inserted into the pGL3-control vector by T4 DNA ligase. The correctly sequenced WT or MUT luciferase reporter plasmids were co-transfected with miR-195-5p mimic into HEK-293T cells. After transfection for 48 h, the cells were collected and lysed. The luciferase activity was detected by the Dual-Luciferase Reporter Assay System kit (Promega Corporation, Madison, WI, USA) on Luminometer TD-20/20 (E5311, Promega Corporation, Madison, WI, USA). The experiment was independently repeated three times.

### Cell culture and selection

The OC cell lines SKOV-3, HO8910, ES-2 and A2780 along with the normal ovarian epithelial cell line IOSE were purchased from the Cell Bank of Shanghai Institute of Cells, Chinese Academy of Science (Shanghai, China). The OC cell lines were cultured in Roswell Park Memorial Institute (RPMI) 1640 medium containing 10% fetal bovine serum (FBS; Gibco, Grand Island, NY, USA), while the IOSE cells were cultured in MCDB105/Medium 199 (Gibco, Grand Island, NY, USA) complete medium. Once the cell confluence reached 80–90%, the cells were detached with 0.25% trypsin and passaged, and cultured in a humidified incubator with 5% CO_2_ in air at 37 °C. The cells at the logarithmic phase of growth were selected for further experiments. At last, the expression of miR-195-5p in different OC cell lines was determined by reverse transcription quantitative polymerase chain reaction (RT-qPCR), and the cell line exhibiting the lowest expression of miR-195-5p was selected for the subsequent assays.

### Cell grouping and transfection

The cells were assigned into the following seven groups: the mimic negative control (NC) group (transfected with NC sequence of miR-195-5p mimic), the miR-195-5p mimic group (transfected with miR-195-5p mimic sequence), the inhibitor NC group (transfected with NC sequence of miR-195-5p inhibitor), the miR-195-5p inhibitor group (transfected with miR-195-5p inhibitor sequence), the mimic NC + over-expressed NC (oe-NC) (transfected with blank control sequence), the miR-195-5p mimic + oe-NC group (transfected with miR-195-5p mimic and blank control sequences), and the miR-195-5p mimic + oe-PSAT1 group (transfected with miR-195-5p mimic and oe-PSAT1 sequences). The transfection sequences in each group are shown in Table 3. The chemically synthesized sequences of mimic NC, miR-195-5p mimic, inhibitor NC, oe-NC and oe-PSAT1 were all purchased from Shanghai GenePharma Co., Ltd. (Shanghai, China). A day prior to transfection, the cells were seeded in a 6-well plate. Once the cell confluence reached 40–60%, liposomes and Lipofectamine™2000 ready for transfection were diluted in serum-free medium, respectively, and completely mixed and allowed to stand for 20 min. Afterwards, the mixture was added into each well and cultured in serum-free medium for 6 h. Following that, the medium was replaced with complete culture medium, and the cells were further cultured for subsequent experiments.

**Table 3:** Gene sequences

Genes	Gene sequence
miR-195-5p mimic NC	5′-ACUACUGAGUGACAGUAGA-3′
miR-195-5p mimic	5′-UAGCAGCACAGAAAUAUUGGC-3′
inhibitor NC	5′-CAGUACUUUUGUGUAGUACAA-3′
miR-195-5p inhibitor	5′-GCCAAUAUUUCUGUGCUGCUA-3′
oe-PSAT1	F: 5′-ATGGACGCCCCCAGGCAGGTG-3′
	R: 5′-AGTATCGACTACGTAGAGGTT-3′

*F* forward, *R* reverse, *NC* negative control, *miR-195-5p* microRNA-195-5p, *oe-PSAT1* overexpressed phosphoserine aminotransferase 1

### Signaling pathway agonist treatment

The β-catenin signaling pathway agonist, WAY262611 (APExBIO, Houston, TX, USA) was dissolved in Dimethyl sulfoxide (DMSO; Sigma, St. Louis, MO, USA) at a final concentration of 2.310 μmol/L [19]. Then, WAY262611 was added to the cells transfected with mimic NC or miR-195-5p mimic sequence. After being cultured for 48 h, the cells were collected for subsequent experiments.

### Cell counting kit-8 (CCK-8) assay

The cells were detached and resuspended, with the concentration adjusted to 1 × 10^5^ cells/mL. Next, the cells were seeded in a 96-well plate with 100 μL/well, and conventionally cultured overnight. DDP with different concentrations (1, 2, 5, 10, 20, and 40 μmol/L) was added to the wells with 5 duplicate wells set for each concentration, and incubated for 48 h. After DDP treatment, the supernatant in each well was discarded and the cells were treated according to the instructions of the CCK-8 kit (Beyotime Biotechnology Co., Ltd., Shanghai, China). Briefly, 10 μL CCK-8 was added to each well, oscillated and further incubated at 37 °C for 1.5 h. The optical density (OD) value of each well at 450 nm was measured using a microplate reader. Subsequently, the inhibition rate was estimated by calculating the percentage of living cells in comparison with the control group. The inhibition rate = (1 − OD_experimental group_/OD_control group_) × 100%. The inhibition rate curve was plotted with the OD values as the ordinate and the DDP concentrations as the abscissa. At last, the semi-inhibition concentration (IC_50_) was calculated using the Probit program of SPSS software.

### Flow cytometry

The OC cells were subdivided into the following 8 groups: the miR-195-5p mimic + saline group (treated with saline); the miR-195-5p mimic + DDP group (final concentration of DDP: 40 μmol/L); the mimic NC + saline group (treated with saline); the mimic NC + DDP group (final concentration of DDP: 40 μmol/L); the miR-195-5p mimic + oe-NC + DDP group (final concentration of DDP: 40 μmol/L); the miR-195-5p mimic + oe-PSAT1 + DDP group (final concentration of DDP: 40 μmol/L); the miR-195-5p mimic + DMSO + DDP group (final concentration of DDP: 40 μmol/L); and the miR-195-5p mimic + WAY262611 + DDP group (final concentration of DDP: 40 μmol/L). After being treated with DDP for 24 h, the cells in each group were rinsed two times with 1 × phosphate buffered solution (PBS) and resuspended with 1 × buffer, with the concentration adjusted to 1 × 10^6^ cells/mL. Subsequently, 100 μL cell suspension was gently mixed with 5 μL Annexin V-fluorescein isothiocyanate (FITC) and 5 μL propidium iodide (PI), incubated at room temperature for 15 min avoiding exposure to light and then added with 400 μL 1 × PBS. At last, the cell apoptosis was detected by flow cytometry using an excitation wavelength of 488 nm.

### Xenograft tumor in nude mice

A total of 48 specific pathogen free (SPF) BALB/c female nude mice (aged 4 weeks; weighing 18–22 g) were randomly grouped. The OC cells were infected with the lentiviral vector expressing agomir NC or miR-195-5p agomir (Shanghai GenePharma Co., Ltd., Shanghai, China). Next, the cells at the logarithmic phase of growth were dispersed into a single cell suspension, with the concentration adjusted to 1 × 10^7^ cells/mL. The cell suspension was subcutaneously inoculated into the right subscapular part of nude mice with 200 μL/mouse to establish xenograft tumor models. When the tumor diameter reached 1 cm, the xenograft tumors in each group were collected and made into 2 mm^3^ tissue blocks. Under aseptic conditions, the tissue blocks were subcutaneously inoculated into the right subscapular part of nude mice. The following nude mice xenograft tumor models were established: the agomir NC group, the miR-195-5p agomir group, the miR-195-5p agomir + saline group, the miR-195-5p agomir + DDP group, the agomir NC + saline group, and the agomir NC + DDP group (8 mice in each group). After being inoculated with xenograft tumors, the nude mice were fed in SPF environment. When the volume of xenograft tumor reached 150 mm^3^, the nude mice were intraperitoneally injected with 2.5 mg/kg DDP or 0.1 mL saline once every 3 days, for a total of six times [20]. The volume of xenograft tumor was measured every 3 days. The maximum diameter (a) and the minimum diameter (b) were measured using Vernier calipers, and the tumor volume was calculated according to the following formula: tumor volume (V) (mm^3^) = π × a×b^2^/6. The growth curve of xenograft tumor was plotted. Subsequently, the nude mice were euthanized 1 week after drug withdrawal. At last, xenograft tumor tissues were dissected, weighed, fixed with 4% paraformaldehyde, paraffin-embedded and sliced into 4 μm serial sections.

### Immunohistochemistry

Immunohistochemical staining was performed using an EliVision™ super kit (mouse/rabbit) (KIT-5220, Maxim Biology, Fuzhou, Fujian, China). Xenograft tumor tissues of nude mice were embedded in paraffin, sectioned and dewaxed. After hydration and antigen thermal repair, the sections were incubated with the primary antibody, mouse anti-human monoclonal antibody to CD34 (KIT-0004, Maxim Biology, Fuzhou, Fujian, China) at 37 °C for 2 h. The primary antibody in the NC group was replaced with PBS. After three PBS rinses (5 min each), the sections were incubated with the secondary antibody, horseradish peroxidase (HRP)-labeled rabbit anti-mouse antibody to IgG at 37 °C for 2 h. Then the sections were rinsed three times with PBS (5 min each), and developed with 3,3′-diaminobenzidine (DAB) (DAB-0031, Maxim Biology, Fuzhou, Fujian, China). Afterward, the sections were counterstained with hematoxylin, rinsed under running water, reacted with hydrochloric–alcohol solution to return to blue. At last, the sections were dehydrated, mounted and observed under an optical microscope. The known positive reaction sections were used as the positive control. Subsequently, the blood vessel-rich “hot spots” areas presented as densely yellowish-brown in xenograft tumor tissues or adjacent tissues of the whole section were identified at 40-fold low power lens. The microvessel density (MVD) was counted under 200-fold visual field using the following criteria: any stained brown-yellow endothelial cell or endothelial cell cluster was recorded as an independent vessel, and the demarcation between each vessel must be clear. A total of five different high-power fields in each section were selected to count the number of vessel and the mean value was obtained. The MVD value obtained was the number of vessels per unit area.

### TdT-mediated dUTP-biotin nick end labeling (TUNEL) staining

The tissue sections of xenograft tumors were fixed with 4% paraformaldehyde, paraffin-embedded and sliced into 4 μm serial sections. Next, the sections were baked at 50 °C for 24 h, dewaxed with xylene, dehydrated with ethanol, and washed with distilled water for 2 min. Then, the sections were detached with 15 μg/mL protease K digestive solution at 37 °C for 15 min, permeated with 0.1% TritonX-100 for 10 min, and incubated with 50 μL TUNEL reaction solution in a wet box at 37 °C for 60 min. A total of 50 μL peroxidase (POD) was added and incubated for 30 min at 37 °C. Subsequently, the sections were incubated with 50 μL DAB color reagent at room temperature for 10 min, mounted with neutral gum and observed under an optical microscope. At last, 10 visual fields were randomly selected in each section with 100 cells counted in each field under the optical microscope. The percentage of apoptotic cell number was calculated as apoptotic index (AI) = apoptotic cell number/total cell number × 100%.

### RT-qPCR

Total RNA was extracted from the fresh frozen OC tissues or transfected cells according to the instructions of the Trizol kit (Invitrogen, Carlsbad, CA, USA). The obtained RNA was treated with RNA-enzyme-free DNA enzyme I, and extracted by phenol and chloroform. Then RNA was dissolved in ultra-pure water treated with diethylpyrocarbonate (DEPC). The OD values of RNA at the wavelengths of 260 nm and 280 nm were measured using a ND-1000 ultraviolet/visible spectrophotometer (Nanodrop Company, Rockford, IL, USA), followed by the determination of quality and concentration of the total RNA. Subsequently, RNA was reverse transcribed into cDNA using the reverse transcription kit. U6 was regarded as the internal reference of miR-195-5p, and β-actin was regarded as the internal reference of other genes. Primer sequences are shown in Table 4. The experiment was independently repeated three times to obtain the mean value.

**Table 4:** Primer sequences for reverse transcription quantitative polymerase chain reaction

Gene	Primer sequence
miR-195-5p	Forward: 5′-CGGGATCCACATCTGGGGCCTTGTGA-3′
	Reverse: 5′-CCCAAGCTTGCTTCGTGCTGTCTGCTT-3′
PSAT1	Forward: 5′-TGCCCAGAAGAATGTTGGCT-3′
	Reverse: 5′-TCCAGAACCAAGCCCATGAC-3′
β-actin	Forward: 5′-GATTCCTATGTGGGCGACGAG-3′
	Reverse: 5′-CCATCTCTTGCTCGAAGTCC-3′
U6	Forward: 5′-CTCGCTTCGGCAGCACA-3′
	Reverse: 5′-AACGCTTCACGAATTTGCGT-3′

*miR-195-5p* microRNA-195-5p, *PSAT1* phosphoserine aminotransferase 1

### Western blot analysis

Total protein was extracted from frozen OC tissues, nude mice xenograft tumor tissues or transfected cells, and the protein concentration of each sample was determined using a bicinchoninic acid (BCA) kit (Thermo Fisher Scientific, Rockford, IL, USA). Next, the proteins were separated by 10% sodium dodecyl sulfate polyacrylamide gel electrophoresis (SDS-PAGE) and transferred onto a nitrocellulose membrane (ZY-160FP, Zeye Bio Co., Ltd., Shanghai, China). The membrane was sealed with 5% skimmed milk for 1 h, and then rinsed three times with tris-buffered saline with tween 20 (TBST; 10 min each). Afterwards, the membrane was incubated with the diluted primary antibodies (dilution ratio of 1:200), rabbit anti-human polyclonal antibodies to PSAT1 (ab96136), hypoxia-inducible factor-1α (HIF-1α; ab51608), vascular endothelial growth factor (VEGF; ab32152), GSK3β (ab32391), p-GSK3β (ab75745), β-catenin (ab32572) and β-actin (ab8226) at 4 °C overnight. All aforementioned antibodies were purchased from Abcam Inc (Cambridge, MA, USA). The following day, the membrane was rinsed three times by TBST (10 min each), incubated with the diluted secondary antibody, HRP-labeled goat anti-rabbit antibody to immunoglobulin G (IgG) polyclonal antibody (dilution ratio of 1:1000, ab, Abcam Inc., Cambridge, MA, USA) at room temperature for 1 h. After being rinsed three times by TBST (10 min each), the membrane was developed with the enhanced chemiluminescence (ECL) solution (ECL808-25, Biomiga Inc, San Diego, USA) at room temperature for 1 min. Then the membrane was photographed with an optical luminescence analyzer (GE Healthcare, Piscataway, NJ, USA), and the relative protein expression was analyzed by gray-scale scanning using Image Pro Plus 6.0 (Media Cybernetics, Bethesda, MD, USA) software with β-actin serving as the internal reference. The experiment was independently repeated three times.

### Statistical analysis

Statistical analyses were processed using the SPSS 21.0 software (IBM Corp. Armonk, NY, USA). All data were tested for normality and homogeneity of variance. Measurement data in line with the normality distribution were expressed as mean ± standard deviation. If the data did not conform to the normal distribution or the homogeneity of variance, data were expressed as interquartile range. Comparison between OC tissues and adjacent normal tissues was carried out using the *t*-test, while skewed data were analyzed by the non-parametric Wilcoxon symbolic rank test. Comparison between multiple groups was analyzed with one-way analysis of variance (ANOVA), followed by the post hoc test. The data at different time points were analyzed by repeated measurement ANOVA. A value of *p* < 0.05 was considered to be indicative of statistical significance.

## Results

### The potential involvement of miR-195-5p and PSAT1 in OC

Microarray analyses were performed to explore the mechanism of miR-195-5p and PSAT1 in OC. The DEGs were screened from OC-related microarray data (GSE54388, GSE40595, GSE38666, GSE18520, GSE14407), with the threshold set as |log2FC| > 2.0 and *adj.P.Val* < 0.05. The top 100 DEGs were selected from each dataset to plot the Venn map (Fig. 1a). A total of 10 intersecting genes were identified (ITLN1, ABCA8, ADH1C, PRG4, OGN, AOX1, REEP1, LGALS2, DFNA5, PSAT1). Simultaneously, the top 10 OC-related genes (BRCA1, TP53, PLOD1, MUC16, BRCA2, VEGFA, ERBB2, FSHR, AKT1, SHBG) were retrieved from the DiGSeE database. The PPI network was constructed using the String database to analyze the interactions between the DEGs and disease genes (Fig. 1b). The results revealed that OGN and PSAT1 were the major DEGs associated with the disease genes. In addition, the heat maps of the top 50 DEGs in GSE54388 and GSE40595 showed that OGN was expressed at low levels in OC tissues while PSAT1 was expressed highly (Fig. 1c, d). Moreover, the expression profiles of PSAT1 in GSE38666, GSE18520 and GSE14407 were extracted. The changes of PSAT1 expression are shown in Fig. 1e–g: PSAT1 was up-regulated in OC. A previous study reported that PSAT1 could regulate the GSK3β/β-catenin signaling pathway, and the inhibition of GSK3β/β-catenin signaling pathway affects the progression of OC [10, 15, 21]. As a result, we speculated that PSAT1 affects OC through the GSK3β/β-catenin signaling pathway. MiRNA-mRNA relationship prediction tools (Target Scan, mirDIP, micropath, miRNA, DIANA, and microSearch) were employed to predict the miRNAs that regulated PSAT1, and Venn diagrams were plotted to compare the prediction results (Fig. 1h). There were two intersecting miRNAs, namely, hsa-miR-16-5p and hsa-miR-195-5p. Interestingly, miR-16 has been previously suggested to serve as a biomarker for the diagnosis and prognosis of OC [22, 23]. However, the significance of miR-195-5p in OC has been seldom studied. Therefore, the current study aimed to validate whether miR-195-5p targeting PSAT1 participates in the development of OC through the GSK3β/β-catenin signaling.

**Fig. 1:** miR-195-5p affects OC progression via PSAT1-mediated GSK3β/β-catenin signaling pathway. **a** Intersection of the top 100 DEGs from datasets GSE54388, GSE40595, GSE38666, GSE18520 and GSE14407; **b** the PPI network of OC-related DEGs and disease genes where the arrow means DEGs, and the circle represents disease genes; **c**, **d** heat map of the top 50 DEGs in GSE54388 and GSE40595, where the abscissa represents the sample number, and the ordinate represents the DEG; upper right histogram is the color gradation where each rectangle corresponds to a sample expression value; **e**–**g** the expression of PSAT1 in datasets GSE38666, GSE18520 and GSE14407. **h** Intersection of predicted miRNAs that target PSAT1 in databases TargetScan, mirDIP, miRopath, microRNA, DIANA and miRSearch

### MiR-195-5p is lowly expressed in OC tissues and cells

The expression of miR-195-5p in OC and adjacent normal tissues was determined by RT-qPCR and the result showed that expression of miR-195-5p in OC tissues was significantly lower than that in adjacent normal tissues (*p *< 0.05; Fig. 2a). In addition, we measured the expression of miR-195-5p in the OC cell lines SKOV-3, HO8910, ES-2, A2780 and the normal ovarian epithelial cell line IOSE (Fig. 2b). It was revealed that the four OC cell lines displayed lower expression of miR-195-5p compared to IOSE cells. In particular, the expression of miR-195-5p in SKOV-3 cells was found to be the lowest among the 4 OC cell lines (*p* < 0.05). Therefore, the OC cell line SKOV-3 was chosen for subsequent experimentation.

**Fig. 2:** miR-195-5p is poorly expressed in OC tissues and cells. **a** Expression of miR-195-5p in adjacent normal tissues (n = 25) and OC tissues (n = 77); **b** expression of miR-195-5p in normal ovarian epithelial cell line and OC cell lines; The above results are regarded as measurement data and represented by mean ± standard deviation; unpaired *t*-test is used for data analysis between two groups, while one-way ANOVA is utilized for data analysis among multiple groups; the experiment was independently repeated three times

### MiR-195-5p inhibits angiogenesis and weakens chemotherapy resistance in OC

The expression patterns of HIF-1α and VEGF in OC tissues were measured by Western blot analysis (Fig. 3a, b). The expression of HIF-1α and VEGF in OC tissues was found to be significantly higher than that in adjacent normal tissues (*p* < 0.05). The OC cells were transfected with miR-195-5p mimic, mimic NC, miR-195-5p inhibitor and inhibitor NC. The changes in the expression of miR-195-5p, HIF-1α and VEGF were identified by RT-qPCR or Western blot analysis (Fig. 3c–e). Compared with the mimic NC group, the expression of miR-195-5p was observed to be significantly increased, and the protein expression of HIF-1α and VEGF was obviously decreased in the miR-195-5p mimic group (all *p* < 0.05). However, the expression of miR-195-5p was significantly inhibited, and the protein expression of HIF-1α and VEGF was higher in the miR-195-5p inhibitor group in comparison with the inhibitor NC group (*p* < 0.05). Taken together, the aforementioned results proved that up-regulation of miR-195-5p could decrease the expression of tumor angiogenesis-related factors in the OC cell line SKOV-3.

**Fig. 3:** Over-expression of miR-195-5p represses angiogenesis and reduces chemotherapy resistance in OC. **a**, **b** Protein expression of HIF-1α and VEGF in adjacent normal tissues (n = 25) and OC tissues (n = 77) detected by Western blot analysis; *p < 0.05 vs. adjacent normal tissues; **c** expression of miR-195-5p in SKOV-3 cells after transfected with corresponding sequences detected by RT-qPCR; *p < 0.05 vs. the mimic NC group; ^#^*p* < 0.05 vs. the inhibitor NC group. **d**, **e** Protein expression of HIF-1α and VEGF in SKOV-3 cells transfected with miR-195-5p mimic or inhibitor measured by Western blot analysis; *p < 0.05 vs. the mimic NC group; ^#^*p* < 0.05 vs. the inhibitor NC group; **f** inhibition rate of SKOV-3 cells at different DDP concentrations after transfection with miR-195-5p mimic or inhibitor evaluated by CCK-8; *p < 0.05 vs. the mimic NC group; **g** IC_50_ value of DDP in SKOV-3 cells after transfected with corresponding sequences detected by CCK-8; *p < 0.05 vs. the mimic NC group; **h**, **i** apoptosis of SKOV-3 cells after transfection with miR-195-5p mimic or inhibitor measured by flow cytometry; *p < 0.05 vs. the mimic NC + saline group; ^#^*p* < 0.05 vs. the mimic NC + DDP group. The above results are measurement data, and expressed as mean ± standard deviation; unpaired *t*-test is used to analyze the data between two groups; while one-way ANOVA is used to analyze the data among multiple groups; the repeated measures ANOVA is performed at different time points; the experiment was independently repeated three times

The drug resistance of OC cells was detected using CCK-8 assay where the cells were transfected with miR-195-5p mimic or mimic-NC after DDP treatment (Fig. 3f, g). The inhibition rate of SKOV-3 cells was found to be promoted with increasing DDP concentration, and the sensitivity of SKOV-3 cells to DDP was increased upon transfection with miR-195-5p mimic. Compared with the mimic NC group, the IC_50_ value of the miR-195-5p mimic group was markedly decreased (*p* < 0.05). Furthermore, the apoptotic rate of the miR-195-5p mimic + DDP group was noted to be significantly increased when compared with the mimic NC + DDP group (*p* < 0.05; Fig. 3h, i). Based on these findings, it can be concluded that up-regulation of miR-195-5p could reduce the chemotherapy resistance.

### MiR-195-5p regulates the GSK3β/β-catenin signaling pathway via inhibition of PSAT1

The expression of PSAT1 in various cancers was retrieved using the bioinformatics website GEPIA (http://gepia.cancer-pku.cn/detail.php?gene=PSAT1). The results revealed that PSAT1 was highly expressed in OC (Fig. 4a). There were miR-195-5p specific binding sites in the 3′UTR of PSAT1, indicating that PSAT1 was the target gene of miR-195-5p. Putative miR-195-5p binding sites on the 3′UTR of PSAT1 were confirmed by dual luciferase reporter gene assay (Fig. 4b). The results displayed that in comparison with the NC group, the luciferase activity was decreased upon co-transfection with the miR-195-5p mimic and PSAT1-3′UTR-WT (*p* < 0.05). However, there were no significant differences in the luciferase activity when co-transfected with the miR-195-5p mimic and PSAT1-3′UTR-MUT (*p* > 0.05). These results verified that miR-195-5p specifically binds to PSAT1 gene and down-regulates its expression.

**Fig. 4:** Over-expression of miR-195-5p restrains PSAT1 and modulates the GSK3β/β-catenin signaling pathway. **a** Predicted expression of PSAT1 in tumor and normal tissues in bioinformatics website GEPIA. **b** Binding of miR-195-5p to PSAT1 predicted by bioinformatics website and verified by dual luciferase reporter gene assay; *p < 0.05 vs. the NC group; **c** mRNA expression of PSAT1 in adjacent normal tissues (n = 25) and OC tissues (n = 77) determined by RT-qPCR; *p < 0.05 vs. the adjacent normal tissues; **d**, **e** protein expression of PSAT1 in adjacent normal tissues (n = 25) and OC tissues (n = 77) detected by Western blot analysis; *p < 0.05 vs. the adjacent normal tissues; **f**, mRNA expression of PSAT1 in SKOV-3 cells when transfected with miR-195-5p mimic or inhibitor detected by RT-qPCR, n = 3; *p < 0.05 vs. the mimic NC group; ^#^*p* < 0.05 vs. the inhibitor NC group. **g**, **h** Protein expression of PSAT1 in SKOV-3 cells when transfected with miR-195-5p mimic or inhibitor detected by Western blot analysis; *p < 0.05 vs. the mimic NC group; ^#^*p* < 0.05 vs. the inhibitor NC group; **i** mRNA expression of PSAT1 in SKOV-3 cells when transfected with miR-195-5p mimic or co-transfected with miR-195-5p mimic and oe-PSAT1 measured by RT-qPCR. *p < 0.05 vs. the mimic NC + oe-NC group; ^#^*p* < 0.05 vs. the miR-195-5p mimic + oe-NC group; **j**, **k** protein expression of GSK3β and β-catenin as well as the extent of GSK3β phosphorylation in SKOV-3 cells when transfected with miR-195-5p mimic or co-transfected with miR-195-5p mimic and oe-PSAT1 measured by Western blot analysis; *p < 0.05 vs. the mimic NC + oe-NC group; ^#^*p* < 0.05 vs. the miR-195-5p mimic + oe-NC group. The above data are measurement data and expressed by mean ± standard deviation; unpaired *t*-test is used to analyze the data between two groups, while one-way ANOVA is used to analyze the data among multiple groups; the experiment was independently repeated three times

The expression of PSAT1 in OC tissues and adjacent normal tissues was determined (Fig. 4c–e). The results displayed that the expression of PSAT1 in OC tissues was significantly higher than that in adjacent normal tissues (*p* < 0.05). Subsequently, the changes in the expression of PSAT1 in OC cells were detected where the cells were transfected with miR-195-5p mimic, mimic NC, miR-195-5p inhibitor or inhibitor NC (Fig. 4f–h). In comparison with the mimic NC group, the expression of PSAT1 was found to be significantly decreased in the miR-195-5p mimic group in comparison with the inhibitor NC group, while that in the miR-195-5p inhibitor group was significantly increased (all *p* < 0.05). Moreover, the expression of PSAT1, GSK3β, and β-catenin and the extent of GSK3β phosphorylation in OC cells were determined by RT-qPCR and Western blot analysis after transfected with mimic NC + oe-NC, miR-195-5p mimic + oe-NC or miR-195-5p mimic + oe-PSAT1 (Fig. 4i–k). In comparison with the mimic NC + oe-NC group, the mRNA expression of PSAT1 was evidently reduced in the miR-195-5p mimic + oe-NC group, as well as the protein expression of β-catenin and the extent of GSK3β phosphorylation (all *p* < 0.05), while the protein expression of GSK3β showed no significant difference (*p* > 0.05). Meanwhile, no significant differences were found in the miR-195-5p mimic + oe-PSAT1 group (*p* > 0.05). Compared with the miR-195-5p mimic + oe-NC group, the miR-195-5p mimic + oe-PSAT1 group displayed significantly increased mRNA expression of PSAT1, protein expression of β-catenin as well as the extent of GSK3β phosphorylation (*p* < 0.05), but the protein expression of GSK3β showed no significant difference (*p* > 0.05). Taken together, the above-mentioned findings suggested that up-regulation of miR-195-5p inhibits the expression of PSAT1 and blocks the activation of GSK3β/β catenin signaling pathway.

### Over-expression of miR-195-5p reduces angiogenesis and chemotherapy resistance by regulating PSAT1 and the GSK3β/β-catenin signaling pathway in OC

The expression of HIF-1α and VEGF was determined by Western blot analysis in OC cells in the miR-195-5p mimic + oe-NC, miR-195-5p mimic + oe-PSAT1, miR-195-5p mimic + DMSO, miR-195-5p mimic + WAY262611 groups (Fig. 5a, b). In contrast to the miR-195-5p mimic + oe-NC group, the expression of HIF-1α and VEGF was noted to be significantly increased in the miR-195-5p mimic + oe-PSAT1 group (*p* < 0.05). The expression of HIF-1α and VEGF in the miR-195-5p mimic + WAY262611 group was markedly enhanced when compared to the miR-195-5p mimic + DMSO group (*p* < 0.05). The above results demonstrated that up-regulation of miR-195-5p inhibits the expression of tumor angiogenesis-related factors in OC cell line SKOV-3 by down-regulating the expression of PSAT1 and blocking the β-catenin signaling pathway.

**Fig. 5:** Over-expression of miR-195-5p represses angiogenesis and chemotherapy resistance in OC via the regulation of PSAT1 and the GSK3β/β-catenin signaling pathway. **a**, **b** Expression of HIF-1α and VEGF in SKOV-3 cells when transfected or treated with miR-195-5p mimic, oe-PSAT1 and WAY262611 (inhibitor of GSK3β/β-catenin signaling pathway); *p < 0.05 vs. the si-NC group; **c** effects of different DDP concentrations on the inhibition rate of SKOV-3 cells when treated with DDP, miR-195-5p mimic, oe-PSAT1 and WAY262611 detected by CCK-8; *p < 0.05 vs. the miR-195-5p mimic + oe-NC group, ^#^*p* < 0.05 vs. the miR-195-5p mimic + DMSO group; **d** IC_50_ value to DDP in SKOV-3 cells after treated with DDP, miR-195-5p mimic, oe-PSAT1 and WAY262611 detected by CCK-8; *p < 0.05 vs. the miR-195-5p mimic + oe-NC group; ^#^*p* < 0.05 vs. the miR-195-5p mimic + DMSO + DDP group; **e**, **f** the apoptosis of SKOV-3 cells when treated with DDP, miR-195-5p mimic, oe-PSAT1 and WAY262611 measured by flow cytometry; *p < 0.05 vs. the miR-195-5p mimic + oe-NC + DDP group; ^#^*p* < 0.05 vs. the miR-195-5p mimic + DMSO + DDP group. The figure data are measurement data and expressed as mean ± standard deviation; one-way ANOVA was used among multiple groups, while repeated measures ANOVA was performed at different time points; the experiment was independently repeated three times

The proliferation of OC cells transfected with miR-195-5p mimic and/or oe-PSAT1 was detected after the treatment of DDP or β-catenin agonist WAY262611 (Fig. 5c, d). The inhibition rate of SKOV-3 cells was noted to be elevated with the increase of DDP concentration. However, the sensitivity of SKOV-3 cells to DDP was decreased after transfection of oe-PSAT1 or treatment with WAY262611. Compared with the miR-195-5p mimic + oe-NC + DDP group, the IC_50_ value in the miR-195-5p mimic + oe-PSAT1 + DDP group was found to be significantly promoted (*p* < 0.05). While the IC_50_ value in the miR-195-5p mimic + WAY262611 + DDP group was significantly increased when compared to the miR-195-5p mimic + DMSO + DDP group (*p *< 0.05). The apoptosis in each group was detected by flow cytometry (Fig. 5e, f). The results revealed the miR-195-5p mimic + oe-PSAT1 + DDP group displayed prominently decreased apoptosis rate compared to the miR-195-5p mimic + oe-NC + DDP group (*p *< 0.05). While the apoptosis rate in the miR-195-5p mimic + WAY262611 + DDP group was significantly lower than that in the miR-195-5p mimic + DMSO + DDP group (*p *< 0.05). Consequently, it could be inferred that up-regulation of miR-195-5p inhibits the activation of PSAT1-dependent GSK3β/β-catenin signaling pathway, thus weakening the chemotherapy resistance.

### Over-expression of miR-195-5p inhibits angiogenesis by impairing the PSAT1-dependent activation of the GSK3β/β-catenin signaling pathway in vivo

The protein expression of PSAT1, GSK3β, β-catenin, HIF-1α and VEGF as well as the extent of GSK3β phosphorylation were determined in the tumors of nude mice (Fig. 6a, b). Compared with the agomir NC group, the protein expression of PSAT1, β-catenin, HIF-1α and VEGF as well as the extent of GSK3β phosphorylation were all found to be repressed in the miR-195-5p agomir group (*p* < 0.05), but the protein expression of GSK3β showed no significant difference (*p* > 0.05). The immunohistochemistry results verified that compared with the nude mice in the agomir NC group, the MVD in xenograft tumors of nude mice in the miR-195-5p agomir group was decreased (*p* < 0.05; Fig. 6c, d). Taken together, these results revealed that over-expression of miR-195-5p blocks the PSAT1-dependent GSK3β/β-catenin signaling pathway and hinders tumor angiogenesis.

**Fig. 6:** Over-expression of miR-195-5p restrains angiogenesis via regulating PSAT1 and GSK3β/β-catenin signaling pathway in vivo. **a**, **b** Protein expression of PSAT1, GSK3β, β-catenin, HIF-1α and VEGF as well as the extent of GSK3β phosphorylation in xenograft tumor of nude mice detected by Western blot analysis; *p < 0.05 vs. the agomir NC group; **c** immunohistochemical staining results in xenograft tumor in nude mice (×400, scale bar = 25 μm). **d** MVD in xenograft tumor in nude mice; *p < 0.05 vs. the agomir NC group. The figure data are measurement data and represented as mean ± standard deviation; one-way ANOVA is used among multiple groups and *t*-test is used between two groups; the experiment was independently repeated three times

### Over-expression of miR-195-5p represses chemotherapy resistance in vivo

Xenograft tumor in nude mice was observed to analyze the effect of miR-195-5p on chemotherapy resistance in vivo. The volume and weight of xenograft tumors were recorded and the growth curve was plotted (Fig. 7a–c). Compared with the agomir NC + DDP group, the volume and weight of xenograft tumors in nude mice were observed to be reduced in the miR-195-5p agomir + DDP group (*p* < 0.05), and compared with the agomir NC + saline group, the volume and weight of xenograft tumors in nude mice of the miR-195-5p agomir + saline group were obviously diminished (*p* < 0.05). TUNEL staining (Fig. 7d, e) revealed that the AI in nude mice was significantly higher in the miR-195-5p agomir + DDP group compared with the agomir NC + DDP group (*p* < 0.05); compared with the agomir NC + saline group, the AI was significantly elevated in the miR-195-5p agomir + saline group (*p* < 0.05). All in all, the findings demonstrated that over-expression of miR-195-5p inhibits the growth of xenograft tumors and reduces the OC cell resistance to DDP.

**Fig. 7:** Over-expression of miR-195-5p inhibits chemotherapy resistance in vivo. **a** The growth curve of xenograft tumors in nude mice; **b** final volume of xenograft tumors; *p < 0.05 vs. the agomir NC + saline group; ^#^*p* < 0.05 vs. the agomir NC + DDP group; **c** final weight of xenograft tumors; *p < 0.05 vs. the agomir NC + saline group; ^#^*p* < 0.05 vs. the agomir NC + DDP group; **d** cell apoptosis of nude mice in xenograft tumors detected by TUNEL staining (×400, scale bar = 25 μm); positive cells are stained as brown-yellow in the nuclei; **e** quantitative apoptosis rate in xenograft tumors of nude mice; *p < 0.05 vs. the agomir NC + saline group; ^#^*p* < 0.05 vs. the agomir NC + DDP group, n = 8 in each group. The figure data are measurement data and expressed as mean ± standard deviation; one-way ANOVA is used among multiple groups and repeated ANOVA is applied at different time points; the experiment was independently repeated three times

## Discussion

OC is a type of fatal gynecological cancer and patients plagued by OC face unsatisfactory diagnoses and poor survival, as a result of OC being asymptomatic in the early stages and a lack of reliable clinical screening methods [24]. Chemotherapy is widely used nowadays; however, majority of OC patients still face the risk of relapse, which is accompanied by high mortality due to the increased resistance to standard chemotherapy based on DDP [25]. Interestingly, miRNAs have been verified to be aberrantly expressed in OC, and may hold vital importance to the development of OC [26]. In particular, miR-195-5p was previously demonstrated to participate in the progression and development of cancer by functioning as a tumor suppressor [27]. The current study aimed to elucidate the effects of miR-195-5p on OC through the GSK3β/β-catenin signaling pathway by targeting PSAT1. Collectively, our findings led to the conclusion that over-expression of miR-195-5p represses the GSK3β/β-catenin signaling pathway via PSAT1 inhibition, thereby hindering angiogenesis and DDP resistance to OC, while promoting apoptosis of OC cells.

Initially, the current study revealed that miR-195-5p was lowly expressed while PSAT1 was highly expressed in OC. Next, employing online prediction software and dual luciferase reporter gene assay, we discovered and verified that PSAT1 was the target gene of miR-195-5p. This specific miR was previously demonstrated to exhibit significantly reduced expression in a study on breast cancer [28]. Furthermore, miR-195-5p is also known to play an anti-tumor role in different human cancers by targeting different genes. For instance, a previous study revealed that miR-195-5p deters osteosarcoma cell proliferation and invasion by inhibiting naked stratum corneum homolog 1 [29]. The tumor-suppressor role played by miR-195 -5p in regulating cell growth and inhibiting cell cycle by targeting cyclin-dependent kinase 8 in colon cancer has also been underscored [30]. Similarly, miR-195-5p operates as an anti-oncogene by targeting PHF19 in hepatocellular carcinoma [31]. In addition, miR-195-5p is known to be lowly expressed in oral squamous cell carcinoma (OSCC), and this reduced expression inhibits OSCC cell apoptosis and promotes cell migration, growth, and invasion [32]. PSAT1, the target gene of miR-195-5p, was previously found to be obviously elevated in non-small cell lung cancer (NSCLC), which prompted NSCLC cell proliferation, cell cycle progression and tumor formation [33]. Up-regulated expression of PSAT1 has also been discovered to be correlated with poor prognoses for nasopharyngeal cancer (NPC) patients [34]. The abovementioned findings are in line with our result that miR-195-5p functions as a tumor suppressor in OC by targeting PSAT1.

In addition, our findings revealed that the expression of HIF-1α, VEGF, β-catenin as well as the extent of GSK3β phosphorylation was reduced after up-regulation of miR-195-5p, suggesting that over-expression of miR-195-5p inhibited angiogenesis and repressed GSK3β/β-catenin signaling pathway. A previous study has verified that HIF-1 wields critical influence on cellular adaptation to alterations in the availability of oxygen [35]. Stabilized HIF-1α transcription complex is also known to be associated with intratumoural hypoxia and over-expressed HIF-1α facilitates tumor metastasis and progression, thereby inducing treatment failure and even death in various cancers [36]. VEGF, a critical mediator of physiological angiogenesis during skeletal growth, embryogenesis and reproductive functions, is known to be involved in pathological angiogenesis induced by intraocular neovascular disorders, tumors and other conditions [37]. Strikingly, angiogenesis repression has been identified as a novel therapeutic method for treating the recurrence or advancement of OC [38]. The over-expression of miR-195 induced the inhibition of angiogenesis by down-regulating the VEGF expression in hepatocellular carcinoma, and might play a similar role in OC [39]. Meanwhile, β-catenin participates in transcriptional modulation and adhesion between cells, and is highly expressed along with GSK3β in OC [40]. Another study further verified that the AKT/GSK3β signaling pathway is correlated with enhanced cell apoptosis and decreased DDP-resistance to OC [41]. These results and findings support that over-expression of miR-195-5p inhibits angiogenesis and represses the GSK3β/β-catenin signaling pathway.

Finally, we uncovered that over-expressed miR-195-5p inhibited angiogenesis and DDP resistance to OC by suppressing PSAT1 and the GSK3β/β-catenin signaling pathway. Angiogenesis has been demonstrated to serve as a therapeutic target for OC treatment [42]. Likewise, miR-199a has been proved to function as a novel biomarker for DDP-resistant OC, which reverses DDP resistance to OC cells [43]. In addition, miR-195 over-expression has been verified to restrain angiogenesis and cell proliferation in human prostate cancer [44]. Also, over-expression of miR-195-5p was previously found to markedly promote CRC cell susceptibility to chemotherapy and accelerate cell apoptosis in chemoresistant CRC cells [45]. Furthermore, inhibition of PSAT1 has been revealed to repress cell proliferation and tumor formation through regulation of the GSK3β/β-catenin signaling pathway in estrogen receptor (ER)-negative breast cancer [10]. Accordingly, these findings and results demonstrate that miR-195-5p inhibits angiogenesis and DDP resistance to OC by suppressing PSAT1 and the GSK3β/β-catenin signaling pathway. The in vivo experiments carried out in our study also verified the inhibitory effect of miR-195-5p on angiogenesis and DDP resistance to OC.

## Conclusion

Taken together, we found decreased miR-195-5p expression in OC, and miR-195-5p could target PSAT1. Finally, we made conclusion that over-expression of miR-195-5p inactivates the GSK3β/β-catenin signaling pathway through suppression of PSAT1, thus inhibiting angiogenesis, reducing chemotherapy resistance of OC to DDP, and promoting OC cell apoptosis, which was also confirmed by in vivo experiments (Fig. 8). However, further investigation involving the mechanism of miR-195-5p, PSAT1 and the GSK3β/β-catenin signaling pathway on OC is warranted to fully uncover their therapeutic value.

**Fig. 8:** Over-expression of miR-195-5p blocks the PSAT1-mediated GSK3β/β-catenin signaling pathway, thus inhibiting angiogenesis and reducing chemotherapy resistance to DDP

## Data Availability

The datasets generated and/or analyzed during the current study are available from the corresponding author on reasonable request.

## Abbreviations

OC: ovarian cancer
EOC: epithelial ovarian cancer
PSAT1: phosphoserine aminotransferase 1
CRC: colorectal cancer
GSK3β: glycogen synthase kinase-3β
GEO: gene expression omnibus
PPI: protein–protein interaction
FIGO: International Federation of Gynecology and Obstetrics
DMEM: Dulbecco’s modified eagle medium
WT: wild-type
MUT: mutant
FBS: fetal bovine serum
RT-qPCR: reverse transcription quantitative polymerase chain reaction
NC: negative control
DMSO: dimethyl sulfoxide
CCK-8: cell counting kit-8
OD: optical density
PBS: phosphate buffered solution
SPF: specific pathogen free
IHC: immunohistochemistry
MVD: microvessel density
DEPC: diethylpyrocarbonate
BCA: bicinchoninic acid
VEGF: vascular endothelial growth factor
ECL: enhanced chemiluminescence
ANOVA: analysis of variance
